The article "Apelin/APJ-Manipulated CaMKK/AMPK/GSK3β Signaling Works as an Endogenous Counterinjury Mechanism in Promoting the Vitality of Random-Pattern Skin Flaps" was published in 2021. Journal: Oxid Med Cell Longev.

# Apelin/APJ-Manipulated CaMKK/AMPK/GSK3*β* Signaling Works as an Endogenous Counterinjury Mechanism in Promoting the Vitality of Random-Pattern Skin Flaps

**DOI:** 10.1155/2021/8836058

**Published:** 2021-01-25

**Authors:** Zhi-Ling Lou, Chen-Xi Zhang, Jia-Feng Li, Rui-Heng Chen, Wei-Jia Wu, Xiao-Fen Hu, Hao-Chun Shi, Wei-Yang Gao, Qi-Feng Zhao

**Affiliations:** ^1^Department of Cardiovascular and Thoracic Surgery, The Second Affiliated Hospital and Yuying Children's Hospital of Wenzhou Medical University, Wenzhou 325000, China; ^2^Children's Heart Center, Institute of Cardiovascular Development and Translational Medicine, The Second Affiliated Hospital and Yuying Children's Hospital of Wenzhou Medical University, Wenzhou 325000, China; ^3^The Second School of Medicine, Wenzhou Medical University, Wenzhou 325000, China; ^4^Department of Orthopaedic Surgery, The Second Affiliated Hospital and Yuying Children's Hospital of Wenzhou Medical University, Wenzhou 325000, China; ^5^Key Laboratory of Orthopaedics of Zhejiang Province, Wenzhou 325000, China; ^6^Zhejiang Chinese Medical University, Hangzhou 310000, China

## Abstract

A random-pattern skin flap plays an important role in the field of wound repair; the mechanisms that influence the survival of random-pattern skin flaps have been extensively studied but little attention has been paid to endogenous counterinjury substances and mechanism. Previous reports reveal that the apelin-APJ axis is an endogenous counterinjury mechanism that has considerable function in protecting against infection, inflammation, oxidative stress, necrosis, and apoptosis in various organs. As an in vivo study, our study proved that the apelin/APJ axis protected the skin flap by alleviating vascular oxidative stress and the apelin/APJ axis works as an antioxidant stress factor dependent on CaMKK/AMPK/GSK3*β* signaling. In addition, the apelin/APJ-manipulated CaMKK/AMPK/GSK3*β*-dependent mechanism improves HUVECs' resistance to oxygen and glucose deprivation/reperfusion (OGD/R), reduces ROS production and accumulation, maintained the normal mitochondrial membrane potential, and suppresses oxidative stress in vitro. Besides, activation of the apelin/APJ axis promotes vascular migration and angiogenesis under relative hypoxia condition through CaMKK/AMPK/GSK3*β* signaling. In a word, we provide new evidence that the apelin/APJ axis is an effective antioxidant and can significantly improve the vitality of random flaps, so it has potential be a promising clinical treatment.

## 1. Introduction

Wound repair is a common clinical problem in surgery. A skin flap has been proven to be one of the most common and effective methods for wound repair in surgical practice. Random-pattern skin flap replantation is increasingly being selected to close large surficial tissue defects caused by various reasons such as trauma, cancer excisions, and congenital deformity corrective surgery [1–3]. Obviously, wound healing is a coordinated, complex process involving oxidative stress, inflammation, cell proliferation, cell migration, and angiogenesis [4]. During skin flap replantation, especially with the purpose of treating large-area wounds, blood supply interruption, oxidative stress, inflammation, and postoperative infection make the distal flap vulnerable to necrosis and to a great extent limit the clinical application of a random skin flap [5–8]. Blood supply recovery is a consequence of vascular stump's initiation, growth, and recanalization from the pedicle to the distal area [3, 9]. During neovascularization, the ischemia-reperfusion injury (IRI) process is inevitable and necessary, in which effective and reasonable artificial intervention can greatly improve the survival of the skin flap by diminishing the accumulation of acute inflammatory cells [10] and suppressing oxidative stress [11]. As it is a main factor resulting from necrosis of grafts [12–14], IRI is frequently targeted by a series of medicine, treatments, and even biomaterials [15–18].

Considering all of the above, discovery of the substances with both proangiogenesis and antioxidant stress may play positive roles in the clinical application of a skin flap. Apelin, a group of peptides initially isolated from the bovine stomach, is an endogenous ligand of the G protein-coupled APJ receptor [19–21]. Only by binding to the APJ receptor could apelin exert their biologic function [19, 22, 23]; while apelin and the APJ receptor are widely distributed in different organs and tissues [22, 23], the apelin/APJ signal axis may play a role in diseases of different organs including pulmonary fibrosis, kidney inflammation [24], acute lung injury (ALI) [25], ischemic heart failure [26], and even osteoporosis [27, 28]. What we are interested in is that the apelin/APJ signal axis is especially related to vascular pathophysiology [24, 29, 30]. In addition, the apelin/APJ axis regulates IRI and antioxidant stress through different mechanisms such as regulating FoxO3 trafficking [31], maintaining the Ca2+ transient [32], attenuating excessive mitochondrial ROS production [21], and restoring the metabolic defects of lipid oxidation [33]. Existing researches lay the foundation for our hypothesis that apelin can be selected as an adjuvant therapy of skin flap transplantation by regulating angiogenesis and treating oxidative stress.

AMP-activated protein kinase (AMPK) is described as the “energy sensor” or “gauge” and expressed in all cell types and is closely related to IRI and oxidative stress. Since a previous study has proven that apelin protected against IRI-involved ROS-mediated inflammation via the AMPK/GSK3*β* pathway activated by apelin receptor/G*α*/PLC/IP3/CaMKK signaling and further upregulated downstream Nrf2-related antioxidant components in the central nervous system [34], skin vessels act as peripheral terminal vessels, and whether a similar mechanism can be established and further improve the survival of a random skin flap is still not clear. Considering this, we carry out our study to verify and increase the feasibility for clinical application. The apelin family is a peptide family, including apelin12, apelin13, apelin17, and apelin36. Our study preliminarily explored the antioxidant stress response and mechanism of the apelin/APJ axis. As a signal axis is damaged under pathological conditions, the apelin/APJ axis has potential therapeutic target value for further research.

## 2. Materials and Methods

### 2.1. Animals and Grouping

6~8-week-old C57BL/6 mice (22-28 g, male) were obtained from the laboratory animal center of Wenzhou Medical University (license no. SCXK [ZJ] 2005-0019). All animal handling procedures (surgery, treatments, and postoperation care) were strictly in accordance with the Guide for the Care and Use of Laboratory Animals of the China National Institutes of Health. All procedures involving mice were approved by the Animal Research Committee of Wenzhou Medical University (wydw2017-0022). Enormous efforts were made to alleviate the pain of the mice during experiments. All mice were housed in standard experimental cages and given free access to food and water at a room temperature of 25°C with a 12 h light/dark cycle. At the beginning of the experiment, 44 C57BL/6 mice were randomly divided into four groups: normal control group (*n* = 8): purely healthy mice without any trauma treatment; random flap group (*n* = 12): treated with 20 *μ*l saline from day 1~day 7 after skin flap operation; random flap+apelin13 group (*n* = 12): treated with apelin13 (50 *μ*g/kg weight) in a volume of 20 *μ*l by tail intravenous injection from day 1~day 7 after skin flap operation; and random flap+apelin13+ML221 group (*n* = 12): treated with apelin13 (50 *μ*g/kg weight) together with ML221 (50 *μ*g/kg weight) in a volume of 20 *μ*l by tail intravenous injection from day 1~day 7 after skin flap operation.

### 2.2. Reagents and Antibodies

Apelin13 (C_69_H_111_N_23_O_16_S, purity ≥ 95%) was bought from Cayman (catalog 2A-13523-1). ML221 (C_17_H_11_N_3_O_6_, purity: 99.25%) was bought from MedChemExpress (CAS. no. 877636-42-5, Shanghai, China). STO-609 (C_19_H_10_N_2_O_3_, purity ≥ 98.0%) was purchased from MedChemExpress (CAS no. 52029-86-4; Monmouth Junction, NJ, USA). Dorsomorphin (compound C: C_24_H_25_N_5_O, purity: 99.65%) was purchased from MedChemExpress (CAS. no. 866405-64-3; Monmouth Junction, NJ, USA). BX795 (C_23_H_26_IN_7_O_2_S, purity: 99.33%) was purchased from MedChemExpress (CAS. no. 702675-74-9; Monmouth Junction, NJ, USA). The primary antibodies against glycogen synthase kinase 3*β* (GSK3*β*), phospho-glycogen synthase kinase 3*β* (p-GSK3*β*) (Ser-9), superoxide dismutase 2 (SOD2), APJ, vascular endothelial growth factor (VEGF), and CD34 were acquired from Proteintech Group (22104-1-AP, 67558-1-Ig, 24127-1-AP, 20341-1-AP, 19003-1-AP, and 14486-1-AP, respectively), and an apelin primary antibody was obtained from Novus Biologicals (H00008862-M01). Primary antibodies against heme oxygenase-1 (HO-1), B-cell-lymphoma-2 (Bcl2), and nuclear factor E2-related factor 2 (Nrf2) were obtained from Abcam (ab13243, ab196495, and ab137550, respectively). Rabbit monoclonal anti-BCL2-associated X (Bax) was purchased from Cell Signaling Technology (Beverly, MA, USA). Secondary antibodies HRP-conjugated AffiniPure goat anti-mouse IgG (H+L), HRP-conjugated AffiniPure goat anti-rabbit IgG (H+L), CoraLite488-conjugated goat anti-mouse IgG (H+L), CoraLite488-conjugated goat anti-rabbit IgG (H+L), CoraLite594-conjugated goat anti-mouse IgG (H+L), and CoraLite594-conjugated goat anti-rabbit IgG (H+L) were purchased from Proteintech Group (SA00001-1, SA00001-2, SA00013-1, SA00013-2, SA00013-3, and SA00013-4, respectively). The Lipid Peroxidation MDA Assay Kit, diamidino-2-phenylindole (DAPI) solution, the BCA Kit, and the BeyoECL Moon Reagent Kit were purchased from Beyotime Biotechnology (Jiangsu, China). IL-1 and TNF*α* detection kits were purchased from Jiancheng Biotechnology (Nanjing, China).

### 2.3. Random Skin Flap Animal Model

Mice were anesthetized with pentobarbital sodium 1% (50 mg/kg, intraperitoneally injection) before operation. An electric shaver and hair removal ointment were used to remove the dorsal fur of mice. Then, a random-pattern, caudal-based skin flap (size: 1.5 × 4.5 cm^2^) was elevated in the mouse dorsum (in the same position in each mouse) beneath the panniculus carnosus as reported previously. The left and right sacral arteries were excised to block bilateral blood supply of the skin flap. By confirming that the blood vessels were amputated, separated flaps were inserted to the original position and sutured with a 7-0 nonabsorbable suture. The random skin area was equally separated into three zones from the pedicle to the distal: proximal (area I), intermediate (area II), and distal (area III) [3, 9].

### 2.4. Cell Culture

The human umbilical vein endothelial cells (HUVECs) are obtained from the American Type Culture Collection (Manassas, VA, USA) and cultured in RPMI 1640 medium containing 10% fetal bovine serum and 1% antibiotics (penicillin, 100 IU/ml; streptomycin, 100 *μ*g/ml) at 37°C at 5% CO_2_ in a constant-temperature incubator.

### 2.5. Oxygen and Glucose Deprivation/Reperfusion (OGD/R) Model

The OGD/R model was established to simulate IRI. HUVECs were cultured in glucose-free and serum-free DMEM containing apelin13 and inhibitors in a hypoxia chamber (Thermo Scientific, USA) containing a gas mixture of 95% N_2_ and 5% CO_2_ for 6 hours; after 6 hours, the medium was replaced by RPMI 1640 medium containing 10% fetal bovine serum, and HUVECs were transferred back to the previous normoxic culture environment for another 6 hours. As for migration and angiogenesis, the culture medium cannot be changed due to the experimental operation; we only arranged a 4-hour short-time glucose oxygen deprivation (OGD) to observe cell migration and tube formation better.

### 2.6. Cell Grouping and Drug Administration

HUVECs were divided into the following groups: normal control group, OGD/R group, OGD/R+apelin13 group, OGD/R+apelin13+ML221 group, OGD/R+apelin13+ STO-609 group, OGD/R+apelin13+DM group, and OGD/R+apelin13+BX795 group. OGD/R+apelin13 group: HUVECs were treated with apelin13 (0.5 *μ*M); OGD/R+apelin13+ML221 group: HUVECs were treated with apelin13 (0.5 *μ*M)+ML221 (0.5 *μ*M); OGD/R+apelin13+STO-609 group: HUVECs were treated with apelin13 (0.5 *μ*M)+STO-609 (0.5 *μ*M); OGD/R+apelin13+DM group: HUVECs were treated with apelin13 (0.5 *μ*M)+DM (50 ng/ml); OGD/R+apelin13+BX795 group: HUVECs were treated with apelin13 (0.5 *μ*M)+BX795 (2 *μ*M); OGD/R+ML221 group: HUVECs were treated with ML221 (0.5 *μ*M); OGD/R+STO-609 group: HUVECs were treated with STO-609 (0.5 *μ*M); OGD/R+DM group: HUVECs were treated with DM (50 ng/ml); OGD/R+BX795 group: HUVECs were treated with BX795 (2 *μ*M); and normal control group: HUVECs were simply treated with saline.

### 2.7. Flap Macroscopic Evaluation

After operation, the viability of skin flaps was tracked macroscopically by necrotic area, edema, colour, and hair conditions on day 1, day 3, and day 7. Then, on day 7, high-resolution photos of the random flaps were obtained to evaluate the viability. All photos were processed by using the Image-Pro Plus imaging software (ver 6.0; Media Cybernetics) to determine the survival area, and the survival percentage of the skin flap was determined as follows: extent of the survival area × 100%/total area (survival and necrotic).

### 2.8. Laser Doppler Blood Flow (LDBF) Measurement

LDBF measurement was performed to evaluate vascular flow and blood supply in whole skin flaps. On day 3, day 5, and day 7, all mice were anesthetized and placed in a warm and quiet room, and the laser Doppler instrument (Moor Instruments, Axminster, UK) was used to scan mice in each group. The infrared Doppler scanning probe scanned the area of the skin flap to record the blood flow distribution as described in the previous literature [3, 9]. Blood flow of the skin flap was visualized with the strong signal (green, yellow, and red shown in pictures) and quantified with Moor LDI Review software (ver 6.1; Moor Instruments). Measurement of each mouse was performed three times at least, and the mean value was used.

### 2.9. Tissue Edema Measurement

Water content reflects edema of the skin flap. As previously described [3, 9], on day 7, skin flap tissue specimens were obtained and weighed and wet weight was recorded. Then, all specimens were dehydrated in an autoclave at a temperature of 50°C and weighed every day; finally, the stabilized weight was recorded as dry weight. The content of water was calculated as follows: percentage of tissue water content = ([wet weight − dry weight]/wet weight) × 100%.

### 2.10. Hematoxylin Eosin (HE) Staining

Skin flap samples (1 cm × 1 cm) of area II were obtained after sacrifice. The extracted skin flap samples were first fixed in 4% paraformaldehyde for 24 hours and then embedded in paraffin wax for transverse sectioning. Sections were sliced at the thickness of 4 *μ*m with a microtome and mounted on adhesion microscope slides (CITOGLAS, Taizhou, China) for HE staining. We calculated the number of microvessels per unit area (1 mm^2^) under a light microscope (Olympus Corp, Tokyo, Japan), which was described as the microvascular density.

### 2.11. Immunohistochemistry (IHC)

Skin flap sections in each group were baked at 65°C for 2 hours, then dewaxed twice in xylene, and hydrated with gradient ethanol baths. After washing, we blocked tissue sections with 3% hydrogen peroxide solution and performed antigen retrieval (20 min, 95°C) with 10.2 mM sodium citrate buffer (pH 6.0). Then, after blocking tissue sections with 10% goat serum albumin phosphate-buffered saline (10 min, 37°C), the sections were incubated with primary antibodies against CD34 (1 : 200), apelin (1 : 200), and APJ (1 : 200) overnight at 4°C. The second day, these sections were incubated with an HRP-conjugated secondary antibody and counterstained with hematoxylin. Finally, these slices were sealed with neutral resin and placed in a ventilation cupboard overnight. Stained flap sections were pictured at ×200 magnification using a DP2-TWAN image-acquisition system (Olympus Corp, Tokyo, Japan). IHC images were evaluated with Image-Pro Plus software (Media Cybernetics) for integral absorbance quantitation of apelin-, APJ-, and CD34-positive blood vessel counting.

### 2.12. Reactive Oxygen Species (ROS) Measurement

HUVECs were cultured on glass creep plates at a seeding density of 1 × 10^5^. After all stimulations, a reactive oxygen species (DCFH-DA) assay kit (Beyotime, China) was used to measure the cellular ROS level according to the manufacturer's instructions. Images were pictured by using an Olympus microscope. The average fluorescence intensity of the fluorescence emitted by DCF is measured by using Image-Pro Plus software, which reflects the accumulation level of ROS in a positive correlation.

### 2.13. Immunofluorescence Staining

HUVECs were cultured on 12-well culture plates containing glass creep plates at a seeding density of 1 × 10^5^. After all stimulations, remove medium and wash creep plates with aseptic phosphate buffer; then, cells were fixed in 4% paraformaldehyde for 20 min and permeabilized with 0.1% Triton X-100 for 20 min. 10% goat serum albumin was used to block plates (10 min, 37°C), and cell creep plates were incubated with primary antibodies against Nrf2 (1 : 200), HO-1 (1 : 200), and SOD2 (1 : 200) overnight at 4°C. For tissue sections, procedures before primary antibody incubation are the same as described in IHC; then, sections were incubated with primary antibodies against apelin (1 : 200) and APJ (1 : 200) overnight at 4°C. The second day, all sections and plates were washed three times with aseptic phosphate buffer, incubated with a CoraLite488/594-conjugated second antibody for 1 hour at 37°C, and finally stained with DAPI. All images were evaluated under a fluorescence microscope (Olympus, Tokyo, Japan). The percentage of Nrf2-, HO-1-, and SOD2-positive cells in the dermal layer was calculated, and apelin- and APJ- positive areas were colocated.

### 2.14. Western Blotting

After being euthanized, samples (0.5 × 0.5 cm) from the middle of area II flaps in each group were removed from mice and stored at −80°C for Western blotting. In vitro, discard the culture medium of each group of cells, wash it with aseptic phosphate buffer, and harvest the cells with cell scrapers on ice. After extracting total protein from the flap tissues and cells with RIPA lysis buffer, protein concentration was measured by using the BCA protein assay kit. An equal amount of 60 *μ*g tissue protein (30 *μ*g cellular protein) was separated by 10-15% gel electrophoresis and transferred to polyvinylidene difluoride membranes (Roche Applied Science, Indianapolis, IN, USA). After blocking with 5% nonfat milk for 2 hours at room temperature, the membranes were incubated with the subsequent primary antibodies at 4°C overnight: VEGF (1 : 1000), CD34 (1 : 1000), APJ (1 : 1000), apelin (1 : 1000), Bcl2 (1 : 1000), Bax (1 : 1000), Nrf2 (1 : 1000), SOD2 (1 : 1000), HO-1 (1 : 1000), t-AMPK (1 : 1000), p-AMPK (1 : 1000), t-GSK3*β* (1 : 1000), p-GSK3*β* (1 : 1000), and GAPDH (1 : 3000). Then, the membranes were incubated with an HRP-conjugated IgG secondary antibody (1 : 1000) for 2 hours at room temperature. The bands on the membranes were imaged using the ECL Moon Reagent Kit. Protein bands' signal intensity was quantified using Image Lab 3.0 software (Bio-Rad, Hercules, CA, USA).

### 2.15. JC-1 Staining

The mitochondrial membrane potential in each group was determined by staining with JC-1 (Beyotime, China) according to the manufacturer's guidelines. Stained cells were observed under a fluorescence microscope (Olympus; Tokyo, Japan).

### 2.16. MDA and Carbonylated Protein Measurements

Cellular lipid peroxidation in each group was measured by using the Lipid Peroxidation MDA Assay Kit (Beyotime, China). Carbonylated protein level was measured by using the Micro Protein Carbonyl Assay Kit (Solarbio, China). All measurements were performed according to the manufacturer's instructions.

### 2.17. Catalase (CAT) and Glutathione (GSH) Measurements

Catalase was measured by using the CAT Assay Kit (Solarbio, China), and GSH was measured by using the GSH Assay Kit (Solarbio, China) according to the manufacturer's instructions.

### 2.18. IL-1 and TNF*α* Measurements

HUVECs were homogenized by using RIPA buffer, and proteins were collected. IL-1 and TNF*α* levels inside HUVEC cells were measured by using, respectively, the IL-1 ELISA kit (Boyun, China) and TNF*α* ELISA kit (Boyun, China) according to the manufacturer's instructions.

### 2.19. Cell Migration and Tube Formation

Transwell assays (8 *μ*m) (Corning, USA) were used to evaluate the HUVECs' migration ability. Briefly, 2 × 10^5^ cells were seeded into the upper chamber in a volume of 200 *μ*l, while the lower chamber contained glucose-free DMEM culture medium (Gibco) with 1% fetal bovine serum (FBS, Gibco) and different components (saline, apelin13, ML221, STO-609, DM, and BX795); then, cells were placed in a hypoxia chamber. Cells treated with RPMI 1640 medium (Meilunbio) with 1% FBS and placed in a normoxic incubator were used as a normal control group. 4 hours after incubation, cells on the upper surface of the upper chamber membrane were carefully wiped off with cotton swabs, fixed in 4% paraformaldehyde for 30 min at room temperature, and then stained with crystal violet to quantify the migrated cells. The migrated cells were pictured using an inverted microscope (Nikon, Japan). A tube formation assay on Matrigel (BD Biosciences, USA) was performed to evaluate the HUVECs' morphogenesis and tube formation capacity. Briefly, Matrigel solution was thawed at 4°C overnight and placed in a *μ*-Slide (10 *μ*l per well, IBIDI, Germany) in a cell incubator for 30 min to solidify. A total of 5000 cells, which were treated with serum-free and glucose-free DMEM culture medium containing different components (saline, apelin13, ML221, STO-609, DM, and BX795), were seeded onto the Matrigel surface and placed in a hypoxia chamber, and cells treated with RPMI 1640 medium with 10% FBS and placed in a normoxic incubator were used as the normal control. Tube formation was observed and quantified under an inverted microscope (Nikon, Japan) after 4 hours.

### 2.20. Statistical Analyses

Statistical analyses and statistical graphs were implemented using GraphPad Prism 8.0 (GraphPad Software, La Jolla, CA, USA). All data are presented as mean ± SD. Comparisons of mean values between two groups were performed using the independent-sample *t*-test. Mean value comparisons among multigroups were performed using one-way ANOVA followed by the Tukey test. *p* < 0.05 was considered significant.

## 3. Results

### 3.1. Apelin and APJ Were Downregulated in Random Skin Flap Tissue

At first, we examined whether the expression of endogenous apelin and its receptor APJ would change in random skin flap tissue. Western blot analysis and immunohistochemistry staining were used to evaluate the expression of apelin and APJ in normal skin tissue and random skin flap tissue. The corresponding results indicated that both apelin and APJ were significantly decreased in random skin flap tissue at day 7 as shown in Figures 1(a) and 1(b). Similarly, compared with normal skin tissue, VEGF, CD34, SOD2, and HO-1 were downregulated synchronously as shown in Figure 1(a). The proapoptotic protein Bax increased while the antiapoptotic factor Bcl2 decreased. Figures 1(c) and 1(d) show the statistical results of Western blot and immunohistochemistry, respectively. Furthermore, the colocalized immunofluorescence double staining of apelin and APJ (Figure 1(e)) in skin vessels showed an appropriate combination of apelin and APJ under normal conditions, which was greatly reduced in a skin flap. After operation, the ability of antioxidative stress of the skin flap decreased and showed an obvious trend of promoting apoptosis.

### 3.2. Apelin13 Protected the Skin Flap from IRI

We tracked the skin flap necrosis status on day 1, day 3, and day 7 after operation in each group and measured tissue edema, and Figures 2(a) and 2(b) suggested that by supplementing with exogenous apelin13 after operation, the necrotic area of the skin flap reduced significantly and skin edema was also much milder. On the contrary, administration of ML221, an inhibitor of APJ, strongly reversed the protective effect of apelin13. Western blot showed that apelin13 enhanced the antioxidative stress ability of the skin flap, upregulated Nrf2, SOD2, and HO-1, promoted better entry to the nucleus of Nrf2, and resisted the apoptosis tendency while ML221 is reversed (Figures 2(h)–2(j)). Laser Doppler scanning imaging reflected the recovery of a vascular bed in the whole area of the random skin flap, and administration of apelin13 visibly promoted the continuation of the vascular stump of the pedicle and wound edge and increased the blood supply of the skin flap (Figures 2(c) and 2(e)). In addition to the positive effect on visible vascular stumps, the apelin13-treated group has richer microvessel distribution than both the random flap group and apelin13+ML221-treated group (Figures 2(f) and 2(g)). Of all the vascular-related indicators, whether it was the abundance of microvessels and the regeneration of vascular stumps, the addition of the inhibitor ML221 made it worst. In addition, apelin protected the random skin flaps from oxidative stress caused by ischemia-reperfusion to a great extent by increasing the level of GSH and CAT; then, oxidative stress marker carbonylated protein level was relatively few (Figure 2(k)).

### 3.3. Apelin13 Protected the HUVECs from OGD/R

As mentioned before, we adopt OGD/R to simulate the IRI after skin flap transplantation. Immunofluorescence and Western blot showed that OGD/R successfully reproduced oxidative stress and apoptosis of the vascular endothelium in vitro. The protective effect of apelin13 on HUVECs was consistent with that in vivo. Apelin13 upregulated Nrf2, SOD2, HO1, and Bcl2, suppressed the expression of Bax, and improved the ability of antioxidant stress and antiapoptosis of HUVECs (Figures 3(a), 3(b), 3(e), and 3(g)). The DCFH-DA fluorescence probe detected a large amount of ROS production and accumulation inside vascular endothelial cells after OGD/R, and treatment with apelin13 helped suppress it and reduced the cell damage caused by ROS during OGD/R (Figures 3(c) and 3(d)). The accumulation of ROS inside cells damages mitochondrial membrane potential and hinders cell energy metabolism. The changes of mitochondrial membrane potential indirectly reflect the state of energy metabolism under oxidative stress. The red and green fluorescence directly revealed the proportion of normal mitochondria. After OGD/R stimulation, mitochondrial membrane potential dropped but apelin13 treatment maintained relatively normal membrane potential (Figures 3(c) and 3(d)). The decrease in mitochondrial membrane potential can be easily detected by the transition of JC-1 from red fluorescence to green fluorescence, which can also be used as an early detection index of apoptosis. Similar to the results of experiments in vivo, GSH and CAT levels were upregulated while carbonylated protein levels were suppressed after apelin13 treatment (Figure 3(f)); thus, the treatment of apelin13 also increased the cellular CAT and GSH and enhanced the ability of vascular endothelial cells to resist OGD/R-induced injury; on the contrary, ML221 reversed the antioxidant function of apelin13.

### 3.4. Apelin13 Activated AMPK/GSK3*β* Signaling In Vivo and In Vitro

In vivo, compared with normal skin tissue, the content of phosphorylated and activated AMPK together with its downstream GSK3*β* phosphorylation ratio decreased significantly in the random flap (Figures 4(a) and 4(b)). We can see that phosphorylated AMPK remains at a high level in the apelin13-treated group, and apelin13 effectively resists the impairment of AMPK phosphorylation involved in IRI of the random flap. While suppressing APJ by ML221, the activation effect of apelin13 on AMPK and GSK3*β* disappeared (Figures 4(c)–4(e)). HUVECs were stimulated by OGD/R in vitro and treated with apelin13 and apelin13+ML221, and we can see that the changes of phosphorylated AMPK and phosphorylated GSK3*β* are consistent with those in vivo (Figures 4(f)–4(h)). AMPK and GSK3*β* played a significant role in protecting the random flap from IRI. This proved once again that there is good consistency between the HUVECs' OGD/R model and the skin flap's IRI.

### 3.5. CaMKK Contributed to Apelin13-Dependent AMPK/GSK3*β* Signaling Activation in HUVECs

The selective and cellular permeable CaMKK inhibitor STO-609 was used to identify the upstream relationship between the G*α* subunit of the G protein-coupled receptor APJ and AMPK after apelin13 activation. By inhibiting CaMKK by STO-609, the phosphorylation activation of downstream AMPK dropped, the phosphorylation of GSK3*β* decreased (Figures 5(a)–5(c)), and the expression antioxidant factors Nrf2, HO-1, and SOD2 decreased (Figures 5(a), 5(f), 5(g), and 5(h)) which largely counteracted the protective effect of apelin. GSH and CAT declined (Figures 5(i) and 5(j)). Oxidative stress marker carbonylated protein (Figure 5(k)), lipid oxidation product MDA (Figure 5(l)), and inflammatory mediators IL-1 and TNF*α* (Figures 5(m) and 5(n)) became much higher in STO-609 treatment groups. At the same time, STO-609 also made the cells show an obvious trend of apoptosis during OGD/R (Figures 5(a), 5(d), and 5(e)).

### 3.6. Dorsomorphin (DM) Blocking Apelin13-Mediated AMPK/GSK3*β*/Nrf2 Signaling Activation in HUVECs

DM is also known as compound C, a selective AMPK inhibitor, which was used to inhibit apelin13-mediated phosphorylation activation of AMPK. Downregulated phosphorylated AMPK led to the decrease in phosphorylated GSK3*β* (Figures 6(a)–6(c)); the same as described before, cellular CAT (Figure 6(i)) and GSH (Figure 6(j)) declined, and the expression levels of antioxidant proteins Nrf2, HO-1, and SOD2 were downregulated parallelly (Figures 6(a), 6(f), 6(g), and 6(h)), which largely counteracted the protective effect of apelin. Accumulation of carbonylated protein (Figure 6(k)), MDA (Figure 6(l)), and inflammatory mediators IL-1 and TNF*α* (Figures 6(m) and 6(n)) increased significantly in DM treatment groups. The inhibition of AMPK by DM also made HUVECs no longer have physiological antiapoptosis ability when they were undergoing OGD/R stimulation (Figures 6(a), 6(d), and 6(e)).

### 3.7. Inhibition of GSK3*β* Phosphorylation Counteracts Apelin13-Induced Nrf2/SOD2 Signaling Activation in HUVECs

BX795 can reduce the phosphorylation of GSK3*β* at Ser9, and GSK3*β* is highly phosphorylated in an inactive configuration under normal physiological conditions. GSK3*β* was activated, and phosphorylation decreased under the stimulation of OGD/R. BX795's inhibition reversed phospho-Ser9-GSK3*β* upregulation mediated by apelin13. BX795 could not reduce phospho-AMPK content obviously (Figures 7(a)–7(c)). BX795 treatment suppressed CAT (Figure 7(i)) and GSH (Figure 7(j)) and downregulated Nrf2, HO-1, and SOD2 (Figures 7(a), 7(f), 7(g), and 7(h)). Synchronously, BX795 treatment aggravated the production and accumulation of carbonylated protein (Figure 7(k)), MDA (Figure 7(l)), and IL-1 and TNF*α* (Figures 7(m) and 7(n)) compared with the apelin13 treatment group. The inhibition of GSK3*β* phosphorylation aggravated oxidative stress inside HUVECs and promoted apoptosis in the pathological environment made by OGD/R (Figures 7(a), 7(d), and 7(e)).

### 3.8. Apelin13 Promoted the Migration of HUVECs and Angiogenesis by CaMKK/AMPK/GSK3*β* Signaling

The migration of vascular endothelial cells is the foundation of angiogenesis. In our study, the Transwell experiment was used to quantify the migrated HUVECs. The tube formation experiment was used to assess the capacity of angiogenesis. When HUVECs are exposed to glucose and oxygen deprivation, both the number of migrated cells and the number of tubes formed decreased visibly. Apelin13 promoted cell migration and tube formation by combining with APJ; contrary to this, ML221 blocked APJ activation and further inhibited apelin13's promotion (Figures 8(a)–8(c)). When we introduced STO-609 into the treatment, apelin13-mediated cell migration and angiogenesis were reversed (Figures 8(d)–8(f)). Similarly, DM inhibiting AMPK phosphorylation (Figures 8(g)–8(i)) and BX795 inhibiting GSK3*β* Ser-9 phosphorylation (Figures 8(j)–8(l)) inhibited cell migration and reduced the tube number in fields. In addition to the antioxidant stress effect mediated by apelin13, CaMKK/AMPK/GSK3*β* signaling also played an important role in promoting HUVEC migration and angiogenic capacity retroactively.

## 4. Discussion

Large-area skin defects caused by severe trauma, burns, tumor resection, and ulcers often need to be repaired by a skin flap, but the occurrence of potential area necrosis limits the scope of the skin flap. Although delayed operation, pressurization, or drug intervention can improve the survival of the skin flap, the survival of the potential area is still different under different interventions and it is still difficult to guarantee the survival of potential areas. So far, there are many studies on promoting the survival of random skin flap transplantation. In order to enhance skin flap viability, a variety of attempts have been made in the postoperation medicine treatment [3], the biomaterial development [7], herbal extract treatment [9], and even acupuncture treatment [35]. However, in clinical application, the curative effect of these methods is not accurate due to potential toxic side effects and unclear therapeutic targets, and many theoretical treatment schemes are not feasible yet. So, it is imperative to further explore its pathogenesis and seek effective therapeutic targets. A random skin flap, lacking a vessel pedicle, and its blood supply mainly come from the regenerated microvessels and small vessel stumps around the wound. It makes ischemia-reperfusion a definite and inevitable pathological process for a random skin flap. Our preexperiments show that the expression abundance of apelin and its receptor APJ decreased in the skin flap after operation. Our study focused on the significant loss of both the orphan receptor APJ and its ligand apelin in the random pattern skin flap. In order to clarify whether apelin plays a protective role in the survival of the skin flap, we try a short-term exogenous apelin supplementation after skin flap operation. The expected result is that the ischemic necrosis of the random skin flap will decrease after apelin treatment. In fact, after apelin treatment, the degree of edema of the flap is reduced, the necrotic area is reduced, and the blood flow signal intensity of LDBF is increased. Our results suggest the administration of exogenous apelin can improve the viability of the skin flap by enhancing the growth of vascular stumps and microangiogenesis in the ischemic area, attenuating oxidative stress and subsequent apoptosis. Fortunately, as we expected and proved, apelin does have both antioxidant stress and angiogenic effects by activating its receptor APJ. We believe that postoperative exogenous supplementation of apelin to awaken the apelin/APJ axis of vessels is a convenient way to ensure the survival of a random flap and apelin is an effective accelerator for flap survival.

It has been proven that apelin attenuates IRI in organs by a variety of mechanisms such as reducing acute injury through suppression of TGF-*β*1 [36], protecting against myocardial IRI by inactivating GSK3*β* [37]. In these studies, the levels of inflammation and oxidative stress are suppressed by apelin. Similarly, our experimental results in vivo showed that the expression of Nrf2, SOD2, and HO-1 decreased, which indirectly reflected the high oxidative stress operation, and the treatment of apelin increased the expression of Nrf2, SOD2, and HO-1 to some extent. In vitro, we stimulated HUVEC cells with OGD/R which was consistent with the ischemia/reperfusion process in vivo to simulate the pathophysiological changes in vessels. Free from any harmful stimulations, the expression of Nrf2 inside cells remained quite satisfying. Immunofluorescence showed a strong signal of Nrf2 in the nucleus. As far as we know, translocation of Nrf2 into the nucleus promotes the expression of ARE-dependent antioxidant genes [38]. As a result, the expression levels of SOD2 and HO-1 increased; in the meantime, the production and accumulation of ROS inside cells were not active and JC-1 staining showed that the mitochondrial membrane potential was not impaired. After OGD/R stimulation, production and accumulation of ROS increased, the content of Nrf2 decreased either at the overall level or in the nucleus, the expression of antioxidant proteins SOD2 and HO-1 was inhibited, and the mitochondrial membrane potential was damaged resulting in the energy metabolic disorder. By treating with apelin13 alone, stimulated HUVECs appeared to have incredible tolerance to OGD/R stimulation, which was manifested in many aspects such as reduction of intracellular ROS, maintenance of intranuclear Nrf2, and a milder mitochondrial membrane potential damage. Given apelin13 treatment together with the inhibitor ML221, apelin13 can no longer activate the APJ receptor as usual, the protective effects were nearly reversed completely, and HUVECs showed a fragile side to OGD/R again.

APJ is an orphan receptor and a G protein-coupled receptor. Apelin13 binds to the APJ receptor and activates it, and the activation of its G*α* subunits (including G*α*i and G*α*q) can activate downstream CaMKK/AMPK/GSK3*β* signaling, then promotes the translocation of Nrf2 into the nucleus, upregulates ARE-dependent antioxidants SOD, NQO1, and HO-1, suppresses oxidative stress, and protects brain and PC12 cells [39]. When the skin tissue is in a normal and healthy state, normal activation of apelin/APJ ensures a proper phosphorylation ratio of AMPK and GSK3*β* which declined in a random flap. As shown in Figure 9, similar to the protective mechanism of the apelin/APJ axis in the brain, treatment with apelin13 restores the phosphorylation ratio of AMPK and GSK3*β* greatly, which means that AMPK/GSK3*β* signaling also exists as a potential protective mechanism in the skin flap in the same way in the brain.

As we all know, the regeneration of vessels and the recovery of blood supply are the essential problems in wound healing. In order to clarify the angiogenesis mechanism, we focus on the activation of apelin/APJ-dependent CaMKK/AMPK/GSK3*β* signaling and the further effect including angiogenesis and antioxidant stress on HUVECs. The selective CaMKK inhibitor STO-609, selective AMPK inhibitor dorsomorphin, and selective GSK3*β* phosphorylation inhibitor BX795 were given to cells separately. BX795 can inhibit Ser9-phosphorylation of GSK3*β* while it cannot change the expression of total GSK3*β* [40]. It is worth noting that phosphorylation of GSK3*β* inactivates GSK3*β* and the maintenance of GSK3*β* activity increases glycogen degradation, glycolysis substrate oxidation, and lactate production, indicating decreased resistance of cells to oxidative stress [41–44]. All these three inhibitors inhibited apelin13's callback of Nrf2, SOD2, and HO-1. The similar changes of metabolite of lipid oxidation MDA and inflammatory mediators IL-1 and TNF*α* were observed, thus reversing apelin13's protective effect on HUVECs. These suggested that apelin13 protected HUVECs from oxidative stress through a CaMKK/AMPK/GSK3*β* signaling-dependent mechanism during OGD/R.

As for the mechanism of angiogenesis, apelin, AMPK, and GSK3*β* have been separately reported to be associated with angiogenesis [45–48]. However, the relationship among apelin, AMPK, and GSK3*β* in angiogenesis has rarely been reported, especially in the environment of ischemia-reperfusion. In view of the fact that apelin13 can protect HUVECs from oxidative stress in vitro, in a CaMKK/AMPK/GSK3*β*-dependent manner after activating the receptor APJ, we are also interested in whether apelin13 promotes angiogenesis in this CaMKK/AMPK/GSK3*β*-dependent manner. Therefore, the model of short-term glucose and oxygen deprivation was established in vitro, and the quantity of migrated cells in Transwell migration assays and tubules' number in tube formation assays were used to comprehensively evaluate angiogenesis capacity. When cells were exposed to OGD, both migrated cells and tubes formed sharply decreased. Apelin13 increased migrated cells and tubes formed. Administration of inhibitors STO-609, dorsomorphin, and BX795 reversed apelin13's angiogenesis promotion; thus, inhibition of CaMKK, AMPK-phosphorylation, and Ser9-phosphorylation of GSK3*β* declined angiogenesis, indicating that apelin13/APJ promoted angiogenesis capacity at least through a CaMKK/AMPK/GSK3*β* signaling-dependent mechanism.

Regarding prospect and deficiency, our study is precisely focused on skin flap vessels. Through this study, we prove that the apelin/APJ signal axis is suppressed in postoperative skin flap vessels, and postoperative supplementation of apelin can not only help skin flap resist the IRI but also promote angiogenesis, ultimately enhancing random skin flap viability through a CaMKK/AMPK/GSK3*β*-dependent mechanism. Apelin is also a kind of widespread inherent polypeptides in animals, which has good compatibility with animals and can effectively reduce the risk of toxicity and side effects. With increasing clinical trials over time, apelin treatment can be expected to be a convenient and efficient clinical application in the field of wound healing. Besides, we also realize that there are still many limitations in our research, and we have yet to show whether apelin/APJ-manipulated CaMKK/AMPK/GSK3*β-*dependent mechanism is the only mechanism of apelin's therapeutic work. Other therapeutic targets of apelin are not known yet. The study focuses on vessels but ignores exploring the function of other tissue components in the skin flap.

## 5. Conclusion

In conclusion, in vivo, our study proved that the apelin/APJ axis protected the skin flap by alleviating vascular oxidative stress and the apelin/APJ axis works as an antioxidant stress factor dependent on CaMKK/AMPK/GSK3*β* signaling. Besides, an apelin/APJ-manipulated CaMKK/AMPK/GSK3*β*-dependent mechanism improves the tolerance of HUVECs to OGD/R, reduces ROS production and accumulation, maintained the normal mitochondrial membrane potential, and suppresses oxidative stress in vitro. It is worth mentioning that activation of the apelin/APJ axis promotes vascular migration and angiogenesis under relative hypoxia condition through CaMKK/AMPK/GSK3*β* signaling. The awakening of the apelin/APJ axis may play a dual role in both antioxidant stress and angiogenesis in wound healing.

## Figures and Tables

**Figure 1:** The apelin/APJ axis was shut down after random flap operation. (a, c) Western blot results of skin tissue suggest that apelin, APJ, CD34, VEGF, SOD2, and HO-1 were significantly downregulated and apoptosis was upregulated (Bcl2 decreased while Bax increased) after random flap operation. (b, d) IHC staining indicated that the apelin- and APJ-positive area almost halved (scale bar: 50 *μ*m). (e) Immunofluorescence colocalization showed that the codistribution of apelin and APJ in skin microvessels decreased significantly after operation (scale bar: 25 *μ*m). The densitometric analysis of all Western blot bands was normalized to GAPDH. *n* = 4 independent experiments. “∗” means compared with the normal control group. ^∗^*p* < 0.05, ^∗∗^*p* < 0.01.

**Figure 2:** Apelin13 treatment promoted the viability of a random flap. (a) Digital photographs of flap appearances of the random flap group, random flap+apelin13 group, and random flap+apelin13+ML221 groups on day 1, day 3, and day 7 and their inner side photos on day 7 were recorded. (b) The percentages of the survival area and edema degree in three groups were quantified and analyzed. (c) Full-field LDBF images of flaps in each group on day 3, day 5, and day 7. (d) A schematic diagram of a rectangular area (1.5 cm × 4.5 cm) of surgery and scanning. (e) The signal intensity of blood flow of flaps was quantified and analyzed. (f) HE staining showed vessels in area II of flaps in all groups (original magnifcation×200; scale bar: 50 *μ*m). IHC staining showed CD34-positive vessels in area II in all groups (original magnification ×200; scale bar: 50 *μ*m). (g) Histogram of mean vessel density and CD34-positive vessel density in each group. Western blot bands of apoptosis indexes (h), antioxidant stress proteins (i), and statistical results (j). The densitometric analysis of all Western blot bands was normalized to GAPDH. Antioxidant enzymes such as CAT and GSH and oxidative marker carbonylated protein levels in all groups of random flaps were measured (k). *n* = 4 independent experiments. “∗” means compared with the normal control group; “#” means compared with the random flap group; “@” means compared with the random flap+apelin13 group. ^∗^*p* < 0.05, ^∗∗^*p* < 0.01.

**Figure 3:** Apelin13 treatment protected the viability of HUVECs against OGD/R. (a, b) Immunofluorescence of Nrf2, HO-1, and SOD2 of HUVECs in all groups (scale bar: 20 *μ*m) and fluorescence intensity quantification. (c, d) Representative images showing ROS levels and JC-1 intensity in the differentially treated and quantified groups. (e) Western blot bands and relative protein levels (Bcl2, Bax, Nrf2, HO-1, and SOD2). (g) The densitometric analysis of all Western blot bands was normalized to GAPDH. (f) CAT, GSH, and carbonylated protein levels in all groups of HUVECs were measured. *n* = 4 independent experiments. “∗” means compared with the normal control group; “#” means compared with the OGD/R group; “@” means compared with the OGD/R+apelin13 group. ^∗^*p* < 0.05, ^∗∗^*p* < 0.01.

**Figure 4:** Apelin13 enhanced random flaps' viability through AMPK/GSK3*β* signaling in vivo and in vitro. (a) Western blot bands suggested phosphorylation difference of GSK3*β* and AMPK between normal skin and random flap. (b) Ratio of phosphorylated AMPK/total AMPK and phosphorylated GSK3*β*/total GSK3*β*. (c–e) Phosphorylation of AMPK and GSK3*β* in all groups after apelin13 with or without ML221 in vivo. (f–h) Phosphorylation of AMPK and GSK3*β* in all groups after apelin13 with or without ML221 in vitro. The densitometric analysis of all Western blot bands was normalized to total protein and GAPDH. *n* = 4 independent experiments. “∗” means compared with the normal control group; “#” means compared with the random flap group (or OGD/R group); “@” means compared with the random flap+apelin13 group (or OGD/R+apelin13 group). ^∗^*p* < 0.05, ^∗∗^*p* < 0.01.

**Figure 5:** Apelin13 protected HUVECs from OGD/R by activating CaMKK-dependent AMPK/GSK3*β* and downstream Nrf2/HO-1/SOD2. (a) Representative Western blot bands of p-AMPK, t-AMPK, p-GSK3*β*, t-GSK3*β*, Nrf2, HO-1, SOD2, Bax, and Bcl2 in different groups. (b–h) Relative expression and phosphorylation ratio. (i–l) CAT, GSH, MDA, and carbonylated protein levels were measured. (m, n) Inflammatory factors IL-1 and TNF*α* measured by using specific detection kits. The densitometric analysis of all Western blot bands was normalized to total protein and GAPDH. *n* = 4 independent experiments. The grouping legends are placed at the bottom of this figure. “∗” means compared with the normal control group; “#” means compared with the OGD/R group; “@” means compared with the OGD/R+apelin13 group; “&” means compared with the OGD/R+apelin13+STO-609 group. ^∗^*p* < 0.05, ^∗∗^*p* < 0.01.

**Figure 6:** DM blocking apelin13-mediated AMPK/GSK3*β*/Nrf2 signaling activation in HUVECs. (a) Representative Western blot bands of p-AMPK, t-AMPK, p-GSK3*β*, t-GSK3*β*, Nrf2, HO-1, SOD2, Bax, and Bcl2 in different groups. (b–h) Relative expression and phosphorylation ratio. (i–l) CAT, GSH, MDA, and carbonylated protein levels were measured. (m, n) Inflammatory factors IL-1 and TNF*α* measured by using specific detection kits. The densitometric analysis of all Western blot bands was normalized to total protein and GAPDH. *n* = 4 independent experiments. The grouping legends are placed at the bottom of this figure. “∗” means compared with the normal control group; “#” means compared with the OGD/R group; “@” means compared with the OGD/R+apelin13 group; “&” means compared with the OGD/R+apelin13+DM group. ^∗^*p* < 0.05, ^∗∗^*p* < 0.01.

**Figure 7:** Inhibition of GSK3*β* Ser-9 phosphorylation counteracts apelin13-induced Nrf2/SOD2 signaling activation in HUVECs. (a) Representative Western blot bands of p-AMPK, t-AMPK, p-GSK3*β*, t-GSK3*β*, Nrf2, HO-1, SOD2, Bax, and Bcl2 in different groups. (b–h) Relative expression and phosphorylation ratio. (i–l) CAT, GSH, MDA, and carbonylated protein levels were measured. (m, n) Inflammatory factors IL-1 and TNF*α* measured by using specific detection kits. The densitometric analysis of all Western blot bands was normalized to total protein and GAPDH. *n* = 4 independent experiments. The grouping legends are placed at the bottom of this figure. “∗” means compared with the normal control group; “#” means compared with the OGD/R group; “@” means compared with the OGD/R+apelin13 group; “&” means compared with the OGD/R+apelin13+BX795 group. ^∗^*p* < 0.05, ^∗∗^*p* < 0.01.

**Figure 8:** Apelin13 enhanced the migration and tube formation of HUVECs under short-time OGD via CaMKK/AMPK/GSK3*β* signaling. (a, d, g, j) Transwell migration assay and tube formation images of HUVECs with different treatments. (b, e, h, k) Statistical histograms of cell migration. (c, f, i, l) Histogram of tube formations in all different groups. *n* = 4 independent experiments. “∗” means compared with the normal control group; “#” means compared with the OGD group; “@” means compared with the OGD+apelin13 group; “&” means compared with the OGD+apelin13+STO-609 or DM and BX795 groups. ^∗^*p* < 0.05, ^∗∗^*p* < 0.01.

**Figure 9:** Potential mechanism underlying the wound healing promotion of apelin13 on IRI-induced skin flap injuries in mice and HUVECs. Apelin13 protected a random-pattern skin flap against IRI-induced oxidative stress and inflammation through AMPK-mediated inhibitory phosphorylation of GSK-3*β* downstream of the G-coupled receptor (APJ), further inducing Nrf2-mediated antioxidant protein expressions and promoting angiogenesis.

## Data Availability

The data used to support the findings of this study are available from the corresponding author upon request.
